The article "Clinical Efficacy of Immunoglobulin Combined with Glucocorticoids in the Treatment of Oculomotor Myasthenia Gravis in Children and the Effect on Serum Immunity" was retracted in 2023. Reasons: signs of a paper mill; suspected computer-generated content; unreliable results or conclusions; lack of ethics approval or compliance.

# Clinical Efficacy of Immunoglobulin Combined with Glucocorticoids in the Treatment of Oculomotor Myasthenia Gravis in Children and the Effect on Serum Immunity

**DOI:** 10.1155/2022/1772881

**Published:** 2022-07-08

**Authors:** Lijun Fan, Yahui Yang, Fan Zhang, Fei Huang

**Affiliations:** ^1^Pediatrics, Hubei Suizhou Central Hospital, Suizhou, Hubei 441300, China; ^2^Pediatrics, Wuhan Hankou Hospital, Wuhan, Hubei 430012, China; ^3^Pediatrics, Hubei Suizhou Maternal and Child Health Hospital, Suizhou, Hubei 441300, China

## Abstract

To investigate the effects of treatment with immunoglobulin on clinical outcomes and immune function in children with oculomotor myasthenia gravis. The clinical data of 100 pediatric patients with oculomotor myasthenia gravis treated in our hospital from January 2019 to December 2021 were selected as the subjects of this retrospective study and divided into a comparison group and a treatment group according to the different treatment methods. The comparison group was treated with glucocorticoids, and the treatment group was treated with immunoglobulin on the basis of the comparison group. The differences in the serum indexes, the effects of immune function, and the clinical efficacy of the two groups were observed and compared. It was found the comparison of immunoglobulin G (IgG), immunoglobulin A (IgA), and immunoglobulin M (IgM) after treatment was significantly different and lower in the treatment group than in the comparison group; the comparison of CD4^+^, CD3^+^, CD4^+^/CD8^+^, and NK cells after treatment was significantly different and higher in the treatment group than in the comparison group. The effective rate of 98.00% in the treatment group was significantly higher than that of 76.00% in the comparison group, and the difference was statistically significant. The clinical efficacy of the two groups showed that the fever, cough, sputum, myasthenia gravis crisis, and gastrointestinal reactions in the treatment group were significantly lower than those in the comparison group. The study indicates that comparative study of children with oculomotor myasthenia gravis treated with immunoglobulin combined with glucocorticoids is more effective, effectively improving the immune level of patients and reducing adverse reactions.

## 1. Introduction

Ocular myasthenia gravis (OMG) is an autoimmune disorder that produces skeletal muscle fatigue due to impaired transmission caused by disruption of postsynaptic membrane acetylcholine receptors (AchR) at the neuromuscular junction (NMJ) [1–3]. OMG starts at a young age, mostly 1-5 years old, and is common in the ocular myasthenia type, combined with thymoma. There is no significant gender difference [4]. Studies have shown that the development of OMG is closely related to autoantibodies, cytokines, and helper T lymphocytes, with Th1 cells acting mainly through the secretion of IL-2, IFN-*γ*, and TNF-*β* [5].

In current clinical treatment, glucocorticoid shock therapy is mainly used for treatment, but long-term and large amounts of hormone medication can disrupt the original metabolic functions of the patient's organism [6]. This leads to an increased incidence of adverse events, so in actual clinical treatment, other drugs are often used in combination with glucocorticoid shock therapy for treatment [7]. This treatment method can improve the therapeutic effect, shorten the treatment time on the one hand, and reduce the amount of glucocorticoids used on the other hand, which in turn reduces the occurrence of adverse events and improves the prognosis [8]. Immunoglobulin is a globulin with a chemical structure with antibody activity, similar to the antibody molecule, and combined treatment with glucocorticoids can effectively deliver antibodies from immunoglobulin to the patient and convert the acetylcholine receptor of immunoglobulin to the patient's own antigen [9]. Thus, it helps the patient's own acetylcholine antibody production and promotes the autoimmune response of the patient's organism, and exogenous IgG can interfere with the binding of AChR antibodies to AChR, thus protecting the ACR from being blocked by antibodies and ultimately playing an immune protective role [10]. Based on this, we have explored the effect of immunoglobulin treatment on the clinical efficacy and immune function of patients with oculomotor myasthenia gravis in children, after treatment with immunoglobulin.

## 2. Material and Methods

### 2.1. Research Object

The clinical data of 100 pediatric patients with oculomotor-type myasthenia gravis treated in our hospital from January 2019 to December 2021 were selected as the subjects of this retrospective study and divided into comparison (*n* = 50) and treatment groups (*n* = 50) according to the difference in treatment methods. Diagnostic criteria: all patients met the diagnostic criteria for oculomotor-type myasthenia gravis in children as described in the Expert Consensus on the Diagnosis and Treatment of Myasthenia Gravis in China [11]; symptoms of generalized weakness, drooping eyes and face, diplopia, dysphagia, chewing weakness, worsening of symptoms after activity, and reduction of symptoms after rest; all symptoms improved after receiving cholinesterase inhibitor treatment.

### 2.2. Include Exclusion Criteria

Inclusion criteria: (1) patients with skeletal muscle weakness, with typical features of aggravation after activity and reduction after rest or “morning lightness and evening heaviness,” positive fatigue test; (2) age 9-12 years, regardless of gender, Osserman's standard typing type I, all cases have not been treated with similar drugs since the onset of the disease; (3) all positive neostigmine test or cholinesterase inhibitor treatment is effective The electromyography showed decreasing amplitude of low-frequency repetitive electrical stimulation without decreasing amplitude of high-frequency waves and/or broadening of single-fiber EMG tremor. Exclusion criteria: (1) patients who are allergic to glucocorticoid drugs, patients who are treated with other immunosuppressive drugs at the same time; (2) patients with severe infectious diseases of other tissues and organs, patients with other malignant neoplasms, etc.; (3) patients who smoke heavily or drink alcohol, patients with coagulation-related diseases, and patients who do not follow medical advice and do not have treatment compliance.

## 3. Methods

In the control group, glucocorticoid therapy was administered by intravenous methylprednisolone 1 g/d for 3 d, followed by oral prednisone 1 mg (kg/d) every morning, and then gradually reduced to a maintenance dose of 5-15 g/qod after the peak of efficacy. If the disease worsens during the reduction process, the dose will be adjusted to the previous dose, and the reduction will be continued after the disease is in remission. In parallel with the dose reduction, the anticholinesterase drug is gradually reduced until it is discontinued. Maintenance doses are usually administered for 6 months or more. Antibiotics are added if there are signs of infection. Oral potassium chloride is given at the same time. Oral prednisone was administered at a dose of 1.0-1.5 mg/kgd (6090 mg/d), which was gradually reduced after peak efficacy, followed by the same methylprednisolone shock therapy. In the treatment group, immunoglobulin therapy was implemented on top of the comparison group with the addition of intravenous gammaglobulin (State Drug Administration S10970081) 0.4 g/(kg-d). The intravenous drip rate of 40 mL/h was maintained at the beginning of the addition, and then, the intravenous drip rate was accelerated every 30 minutes by 10 mL/h each time, up to 100 mL/h.

### 3.1. Observation Indicator

(1) Humoral immune indexes (immunoglobulin gG, gA, gM, complement C3, and C4), cellular immune indexes (T lymphocyte subpopulation and NK cells). (2) Clinical efficacy: cure: muscle strength recovered, stop using drugs; improvement: muscle strength recovered significantly, related symptoms relieved significantly, muscle strength recovered to some extent, and related symptoms relieved to some extent; invalid: muscle weakness and clinical symptoms did not change, efficiency = (cure + improvement) − 100%.

### 3.2. Statistical Analysis

All statistical data in this study were entered into excel software by the first author and the corresponding author, respectively, and the statistical processing software was SPSS25.0 for calculation. Repeated measures analysis of variance between groups was used to measure the measurement expressed as mean ± standard deviation (*X* ± *S*). Count data expressed as a percentage (%) were tested by *χ*^2^. the risk factors with significant differences were screened. Included data that did not conform to a normal distribution were described by *M*(QR), using the Mann–Whitney test. The statistical significance was *P* < 0.05.

## 4. Results

### 4.1. Comparison of General Data

There was no statistically significant difference between the two groups by *t*-test and chi-square test (*P* > 0.05) in the comparison of general data such as gender, mean age, mean disease duration, and mean weight of patients, see Table 1.

### 4.2. Comparison of Humoral Immunity Levels

Before treatment, there was no significant difference in the humoral immunity levels between the two groups before treatment (*P* > 0.05), but the differences in IgG, IgA, and IgM after treatment were significant, and the treatment group was lower than the control group, with statistical significance (*P* < 0.05), while there was no significant difference in complement C3 and C4 between the two groups (*P* > 0.05), see Figure 1.

### 4.3. Comparison of Cellular Immunity Levels

There was no significant difference in the immune level between the two groups before treatment (*P* > 0.05), but the CD4+, CD3+, CD4+/CD8+, and NK cells after treatment were significantly different, the treatment group was higher than the control group, and the comparison was statistically significant (*P* < 0.05), see Figure 2.

### 4.4. Comparison of Clinical Efficacy and Complications

The effective rate of the treatment group, 98.00%, was significantly higher than that of the control group, 76.00%, and the difference was statistically significant (*P* < 0.05). The clinical efficacy of the two groups of patients showed that the fever, cough, expectoration, myasthenic crisis, and gastrointestinal reactions in the treatment group were significantly lower than those in the control group, and the differences were statistically significant (*P* < 0.05), see Figure 3.

## 5. Discussion

Myasthenia gravis, as an acquired autoimmune disease of the nervous system, can involve the skeletal muscles of the whole body and even the pharyngeal and respiratory muscles, which can endanger the life of patients in severe cases [12]. While the pathogenesis of myasthenia gravis is still unclear in clinical practice, the clinical treatment is also drug-based, and glucocorticoid shock therapy is mainly used in current clinical treatment [13]. The development of dependence on glucocorticoids affects the normal acetylcholine receptor activity in the patient's organism, causing more adverse reactions in patients and leading to myasthenia gravis crisis [14]. Therefore, the treatment of patients with myasthenia gravis requires the selection of safer and more effective treatment modalities. Currently, immunoglobulin has become a common drug used in clinical medicine in combination with glucocorticoid shock therapy, which can effectively enhance patients' autoantibody competition through intravenous immunoglobulin infusion [15]. And using the patient's own negative feedback mechanism to inhibit plasma cell production of antibodies in vivo and promote the elimination of immune complexes in patients can effectively relieve patients' muscle weakness symptoms in the short term [16].

The comparison of IgG, IgA, and IgM after treatment in our study was significantly different and lower in the treatment group than in the comparison group, and the comparison was statistically significant, while there was no significant statistical difference in the comparison of complement C3 and C4 between the two groups. It indicates that immunoglobulin injection has an important role in improving the immune function of the patient's organism, and intravenous immunoglobulin has a fast onset of action, no long-term toxic side effects, and its dose can be reduced when used in combination with glucocorticoids. It was found that the symptoms of OMG patients improved to varying degrees after the application of immunoglobulin, and most patients began to improve their symptoms within 45 d of starting treatment, and the efficacy lasted for about 2 months [17]. In addition, intravenous immunoglobulin does not require placement of a central venous cannula and is well tolerated, with only minimal and mild side effects, making it safer and more reliable for elderly patients or patients with hypotension and neurological disorders [18]. The relationship between complement and MG is also receiving increasing attention, as it plays an important role in the pathogenesis of OMG, with C3 and C4 forming a membrane attack complex deposited at the NMJ, thereby disrupting AChR transmission [19]. OMG patients and EAMG contain an activated fragment of C3 at the NMJ, and complement activation at the NMJ is the initial cause of AChR loss and failure of neuromuscular transmission [20]. Low expression of intrinsic complement regulators in extraocular muscles makes them more sensitive to complement-mediated injury [21]. Some studies have suggested the presence of C3 and C4 depletion in OMG patients, while others have found reduced serum C3 in OMG patients [22]. The role of complement in the pathogenesis of OMG is receiving increasing attention, as antigen-antibody complexes can activate the complement system via the classical pathway due to the presence of autoantibodies, causing autoimmune diseases [23]. Because the condition of OMG patients is the result of a combination of multiple factors, it is not yet possible to explain all patients with one causative factor; multiple complement components interact with each other, other factors synergistically lead to the development of OMG, and complement concentrations may also be influenced by a variety of other factors, so the correlation between C3, C4, and the condition may be poor [24].

The differences in CD4+, CD3+, CD4+/CD8+, and NK cell comparisons after treatment in our study were significant and higher in the treatment group than in the comparison group, and the comparisons were statistically significant. cd4+ lymphocytes are the phenotype of T helper cells that function primarily to assist and induce the generation of the immune response [25]. CD8+ lymphocytes, as a subpopulation of suppressive (Ts) or cytotoxic (Tc) lymphocytes, have a suppressive regulatory function on the immune response [26]. Previous studies have shown10,that patients with OMG have an increased ratio of CD4+ T lymphocytes, a decreased ratio of CD8+ lymphocytes, an increased CD4/CD8+ ratio, and an imbalance in cellular immune regulation, leading to hyperimmune function [27]. Autoimmune tolerance is disrupted, resulting in the production of antibodies against autoantigens causing autoimmune damage [28]. NK cells are an important component of the innate immune system and have the function to defend against infection and prevent malignant transformation of cells [29]. It has been found that peripheral blood NK cell activity is significantly lower in patients with OMG than in normal subjects, and the reduced percentage of NK cells in the blood may be one of the reasons for the immune disorders that occur in OMG producing AchRab, and thus causing pathological damage [30]. Causes of CD4+ and CD8+ ratio dysregulation: it was found that T lymphocytes in the peripheral blood of OMG patients are impaired in regulation and are predominantly impaired in apoptosis of CD4+ T cells, and the dysregulation of CD4+ and CD8+ ratio may be related to this [31]. Due to impaired apoptosis of CD4+ T lymphocytes, activated self-reactive T cells cannot be cleared in a timely manner, and activated T cells cause B cells to proliferate by leaps and bounds, causing an overpowering immune response and the production of antibodies against autoantigens, which leads to the development of autoimmune diseases such as OMG [32].

In our study, the effective rate of 98.00% in the treatment group was significantly higher than that of 76.00% in the comparison group, and the difference was statistically significant. The clinical efficacy of the two groups of patients showed that the fever, cough, sputum, myalgias crisis, and gastrointestinal reactions in the treatment group were significantly lower than those in the comparison group, and the difference was statistically significant by test. Some medical experts believe that among the treatment options, glucocorticoid shock therapy is still the primary choice of clinical treatment, and glucocorticoids can inhibit the activity of lymphocytes in patients, suppress their proliferation and activation, and reduce the release of inflammatory cytokines [33]. Glucocorticoid shock therapy can achieve significant stimulation of lymphocyte activity in the patient's organism in the short term and effectively relieve the clinical symptoms of patients [34]. However, for the higher dosage present in the treatment may lead to more pronounced symptoms of muscle weakness in patients and the occurrence of adverse events such as nausea and dizziness, so in order to reduce the adverse events and improve the actual efficacy of glucocorticoid therapy with high doses [35], the combination of intravenous immunoglobulin infusion and glucocorticoid shock therapy was used with the aim of, on the one hand, giving full play to glucocorticoids to regulate immune function, inhibit choline acetate receptor antibody production, and further repair the motor endplates of the neuromuscular junction [36]. On the other hand, intravenous immunoglobulin was used to regulate the cellular and humoral immune functions of patients, neutralize the AChR antibodies that cause the occurrence of myasthenia gravis, thereby protecting the target tissues of patients, improving the clearance of their autoimmune complexes, reducing the occurrence of adverse events after the use of glucocorticoid shock therapy, and guaranteeing the effectiveness and safety of treatment [37].

Our study is novel but deficient in that the clinical efficacy of replacement immunoglobulin glucocorticoid therapy in children with oculomotor myasthenia gravis is significant, but the specific mechanism has not been studied in depth for a long time. The cases collected from the same hospital were poorly represented, and both exclusion and inclusion were subjective, which may lead to biased results. In conclusion, the comparative study of oculomotor type myasthenia gravis in children treated with immunoglobulin combined with glucocorticoids was more effective, which effectively improved the immune level of patients and reduced adverse reactions, providing some reference value for clinical treatment of oculomotor type myasthenia gravis in children.

## Figures and Tables

**Figure 1:** Comparison of humoral immunity levels (the data related to the comparison of humoral immunity levels of the patients included in our study are expressed as mean ± standard deviation (*X* ± *S*)).

**Figure 2:** Comparison of cellular immunity levels (the data related to the comparison of cellular immunity levels of the patients included in our study were expressed as mean ± standard deviation (*X* ± *S*)).

**Figure 3:** Comparison of clinical efficacy and complications (the clinical efficacy and complication-related data of the patients included in our study were expressed as integers).

**Table 1:** Comparison of general information between the two groups (*n*, $\bar{x}\pm \text{s}$).

Group	Gender (male/female)	Average age (years)	Average duration of illness (months)	Patient weight (kg)
Comparison group (50)	12/38	7.78 ± 1.32	11.34 ± 3.25	43.34 ± 0.25
Treatment group (50)	11/39	7.62 ± 1.66	11.31 ± 3.64	43.31 ± 0.64
*χ* ^2^/*t*	0.056	0.533	0.043	0.309
*P*	0.812	0.595	0.965	0.758

## Data Availability

The datasets used and analyzed during the current study are available from the corresponding author upon reasonable request.

## References

[1] Widemouthed M., Junger D., Leitritz M. A., Neumann J., Neumuth T., Burgert O. (2017). Application fields for the new object management group (OMG) standards case management model and notation (CMMN) and decision management notation (DMN) in the perioperative field. *International Journal of Computer Assisted Radiology and Surgery*.

[2] Feng X., Huan X., Yan C. (2020). Adult ocular myasthenia gravis conversion: a single-center retrospective analysis in China. *European Neurology*.

[3] Witthayaweerasak J., Rattanalert N., Aui-Aree N. (2021). Prognostic factors for conversion to generalization in ocular myasthenia gravis. *Medicine (Baltimore)*.

[4] Akan O., Baysal-Kirac L. (2021). Ophthalmologic manifestations in myasthenia gravis: presentation and prognosis. *Acta Neurologica Belgica*.

[5] Lorenzo C. J., Fitzpatrick H., Campdesuner V., George J., Lattanzio N. (2020). Pembrolizumab-induced ocular myasthenic crisis. *Cureus*.

[6] Li M., Ge F., Guo R. (2019). Do early prednisolone and other immunosuppressant therapies prevent generalization in ocular myasthenia gravis in Western populations: a systematic review and meta-analysis. *Therapeutic Advances in Neurological Disorders*.

[7] Deymeer F. (2020). Myasthenia gravis: MuSK MG, late-onset MG and ocular MG. *Acta Myologica*.

[8] Verma R., Wolfe G. I., Kupersmith M. J. (2021). Ocular myasthenia gravis - how effective is low dose prednisone long term?. *Journal of the Neurological Sciences*.

[9] Hartmann B., Müller M., Seyler L. (2021). Feasibility of deuterium magnetic resonance spectroscopy of 3-O-methylglucose at 7 Tesla. *PLoS One*.

[10] Nagaishi A., Narita T., Woodhall M. (2021). Autoantibodies in Japanese patients with ocular myasthenia gravis. *Muscle & Nerve*.

[11] Neuroimmunology Group of Neurology Branch of Chinese Medical Association, Neuroimmunology Branch of Chinese Society of Immunology (2011). Expert consensus on diagnosis and treatment of myasthenia gravis in China. *Chinese Journal of Neuroimmunology and Neurology*.

[12] Vaphiades M. S., Bhatti M. T., Lesser R. L. (2012). Ocular myasthenia gravis. *Current Opinion in Ophthalmology*.

[13] Wu Y. J., Yan L., Hu Y. X. (2019). Research advances in ocular myasthenia gravis. *Zhongguo Yi Xue Ke Xue Yuan Xue Bao*.

[14] McHugh M. C., Saperstein S. L., Gold R. S. (2019). OMG U #cyberbully! An exploration of public discourse about cyberbullying on twitter. *Health Education & Behavior*.

[15] Lilo E. A., West A. (2021). "OMG, I get like 100 teaspoons of sugar a day!" Rural teens' grasp of their beverage consumption habits. *International Quarterly of Community Health Education*.

[16] Rosenberg H., Ophir Y., Billig M. (2021). OMG, R U OK? Therapeutic relationships between caregivers and youth at risk on social media. *Children and youth services review*.

[17] Graff-Dubois S., Sibéril S., Elluru S. (2007). Use of intravenous polyclonal immunoglobulins in autoimmune and inflammatory disorders. *Transfusion Clinique et Biologique*.

[18] Debus J., Lemaire P., Alani M. (2018). Lymphoplasmacytic lymphoma or multiple myeloma: immunoglobulins may lead to misdiagnosis. *Annales de Biologie Clinique*.

[19] Peter J. G., Chapel H. (2014). Immunoglobulin replacement therapy for primary immunodeficiencies. *Immunotherapy*.

[20] Quast I., Lünemann J. D. (2014). Fc glycan-modulated immunoglobulin G effector functions. *Journal of Clinical Immunology*.

[21] Caner I., Koca E., Ozdemir O. (2021). Serum levels of immunoglobulin isotypes and immunoglobulin g subtypes in healthy term Turkish newborns. *Nigerian Journal of Clinical Practice*.

[22] Lee L., Samardzic K., Wallach M., Frumkin L. R., Mochly-Rosen D. (2021). Immunoglobulin Y for potential diagnostic and therapeutic applications in infectious diseases. *Frontiers in Immunology*.

[23] Abdelhafidh N. B., Toujeni S., Kefi A. (2016). Dermatomyosite et panniculite: place des immunoglobulines [dermatomyositis and panniculitis: the function of immunoglobulins]. *Pan African Medical Journal*.

[24] Lundqvist M. L., Middleton D. L., Radford C., Warr G. W., Magor K. E. (2006). Immunoglobulins of the non-galliform birds: antibody expression and repertoire in the duck. *Developmental and Comparative Immunology*.

[25] Esen F., Senturk E., Ozcan P. E. (2012). Intravenous immunoglobulins prevent the breakdown of the blood-brain barrier in experimentally induced sepsis. *Critical Care Medicine*.

[26] López-Requena A., Mateo De Acosta C., Vázquez A. M., Pérez R. (2007). Immunogenicity of autologous immunoglobulins: principles and practices. *Molecular Immunology*.

[27] Liu X., Cao W., Li T. (2020). High-dose intravenous immunoglobulins in the treatment of severe acute viral pneumonia: the known mechanisms and clinical effects. *Frontiers in Immunology*.

[28] Kurz M. (2008). Developing therapeutic Immunoglobulins. *BioDrugs*.

[29] Yehudai D., Vadasz Z. (2012). IgM enriched immunoglobulins as a therapy for sepsis and autoimmune diseases. *Harefuah*.

[30] Olivieri D. N., Garet E., Estevez O., Sánchez-Espinel C., Gambón-Deza F. (2016). Genomic structure and expression of immunoglobulins in squamata. *Molecular Immunology*.

[31] Guptill J. T., Juel V. C., Massey J. M. (2016). Effect of therapeutic plasma exchange on immunoglobulins in myasthenia gravis. *Autoimmunity*.

[32] Puppel K., Gołębiewski M., Slósarz J. (2021). Interaction between the level of immunoglobulins and number of somatic cells as a factor shaping the immunomodulating properties of colostrum. *Scientific Reports*.

[33] Melamed I., Testori A., Spirer Z. (2012). Subcutaneous immunoglobulins: product characteristics and their role in primary immunodeficiency disease. *International Reviews of Immunology*.

[34] Surace S. J., Deitch J., Johnston R. V., Buchbinder R. (2020). Shock wave therapy for rotator cuff disease with or without calcification. *Cochrane Database of Systematic Reviews*.

[35] Petersen T., Mahévas T., Cannet P. (2021). IgG1 subclass restriction and biochemical peculiarities of monoclonal immunoglobulins in scleromyxedema. *Clinical Laboratory*.

[36] Bermejo-Martin J. F., Giamarellos-Bourboulis E. J. (2015). Endogenous immunoglobulins and sepsis: new perspectives for guiding replacement therapies. *International Journal of Antimicrobial Agents*.

[37] Ermakov E. A., Nevinsky G. A., Buneva V. N. (2020). Immunoglobulins with non-canonical functions in inflammatory and autoimmune disease states. *International Journal of Molecular Sciences*.

